# Distinct Pathways of ERK1/2 Activation by Hydroxy-Carboxylic Acid Receptor-1

**DOI:** 10.1371/journal.pone.0093041

**Published:** 2014-03-26

**Authors:** Guo Li, Hui-qian Wang, Li-hui Wang, Ru-ping Chen, Jun-ping Liu

**Affiliations:** Institute of Aging Research, School of Medicine, Hangzhou Normal University, Hangzhou, Zhejiang, China; University of Louisville, United States of America

## Abstract

Mechanistic investigations have shown that, upon agonist activation, hydroxy-carboxylic acid receptor-1(HCA_1_) couples to a G_i_ protein and inhibits adenylate cyclase activity, leading to inhibition of liberation of free fatty acid. However, the underlying molecular mechanisms for HCA_1_ signaling remain largely unknown. Using CHO-K1 cells stably expressing HCA_1_, and L6 cells, which endogenously express rat HCA_1_ receptors, we found that activation of ERK1/2 by HCA_1_ was rapid, peaking at 5 min, and was significantly blocked by pertussis toxin. Furthermore, time course experiments with different kinase inhibitors demonstrated that HCA_1_ induced ERK1/2 activation via the extracellular Ca^2+^, PKC and IGF-I receptor transactivation-dependent pathways. In addition, we observed that pretreated the cells with M119K, an inhibitor of G_βγ_ subunit-dependent signaling, effectively attenuated the ERK1/2 activation triggered by HCA_1_, suggesting a critical role for βγ-subunits in HCA_1_-activated ERK1/2 phosphorylation. Furthermore, the present results also indicated that the arrestin2/3 were not required for ERK1/2 activation. In conclusion, our findings demonstrate that upon binding to agonist, HCA_1_ receptors initially activate G_i_, leading to dissociation of the G_βγ_ subunit from activated G_i_, and subsequently induce ERK1/2 activation via two distinct pathways: one PKC-dependent pathway and the other IGF-IR transactivation-dependent pathway. Our results provide the first in-depth evidence that defines the molecular mechanism of HCA_1_-mediated ERK1/2 activation.

## Introduction

The G-protein-coupled receptor family includes members that mediate specific actions of hydroxyl carboxylic acids (HCA). HCA_1_ (GPR81) is endogenously activated by lactate [1], HCA_2_ (GPR109A) by 3-hydroxy-butyrate [2], and HCA_3_ (GPR109B) by 3-hydroxylated β-oxidation intermediates, especially 3-hydroxy-octanoic acid [3]. All three receptors couple to G_i_ proteins [4]. The HCA_1_ is prominent in adipose tissue [1], [5], [6], but it is known also to be expressed in a wider range of organs such as liver, kidney and skeletal muscle [1]. In addition, expression of HCA_1_ was increased during differentiation of 3T3-L1 preadipocytes [1], [6]. Unlike HCA_2_, HCA_1_ was not found to be expressed in Langerhans cells or other immune cells in the skin. Activation of HCA_1_ in adipocytes by lactate results in the inhibition of lipolysis at physiologically relevant lactate concentrations (1 to 20 mM) [1], suggesting that HCA_1_ could be a new target for dyslipidemia treatment without the unwanted side effect of cutaneuous flushing.

Almost all GPCRs signal through the mitogen-activated protein kinase (MAPK) cascades, which are traditionally associated with growth factor receptor signaling and are involved in the control of cell proliferation and growth [7], mobility [8], differentiation [9] and apoptosis [10]. Previous studies demonstrated that activation of HCA_1_ by lactate evoked phosphorylation of ERK1/2 in a pertussis toxin-sensitive way [1]. However, the precise mechanism of HCA_1_-mediated ERK1/2 activation remains largely unknown. It has been suggested that lactate plays a role in insulin signaling, particularly in insulin mediated anti-lipolytic effects. It has also been suggested that HCA_1_ may play a role in muscle glucose and fatty acid metabolism. Moreover, a recent study has indicated palmitic acid acutely stimulates glucose uptake via activation of Akt and ERK1/2 in skeletal muscle cells [11]. Therefore, further elucidation of ERK1/2 activation via HCA_1_ will be important for understanding the molecular mechanism for HCA_1_ in the regulation of anti-lipolytic effect and glucose and fatty acid metabolism.

In the present study, we used three cellular backgrounds to characterize the mechanistic details of coupling of the human HCA_1_ to the ERK1/2 signaling pathway: CHO-K1 and HEK293 cells, which recombinantly express human HCA_1_ receptors; and L6 cells, a rat skeletal muscle cell line, which endogenously express rat HCA_1_ receptors. We document here, for the first time, the molecular mechanisms underlying the coupling of the human HCA_1_ to the ERK1/2 MAP kinase pathway in CHO-K1 and L6 cells and implicate the G_i_ protein-initiated PKC and IGF-I receptor transactivation-dependent pathways. Furthermore, using arrestin-2/3 specific siRNA, arrestin-2 and arrestin-3 are found to play no role in HCA_1_-mediated ERK1/2 activation, whereas HCA_1_ internalization is arrestin3-dependent. Our results provide the first in-depth evidence that defines the molecular mechanism of HCA_1_-mediated ERK1/2 activation.

## Materials and Methods

### Materials

Lipofectamine 2000 and G418 were purchased from Invitrogen (Carlsbad, CA). Cell culture media and fetal bovine serum was obtained from Hyclone (Beijing, China). Pertussis toxin (PTX), Go6983, GF109203X (bisindolymaleimide), and tyrphostin A9 were purchased from Sigma (St. Louis, MO). Anti-α-tubulin antibody and RIPA lysis buffer were obtained from Beyotime (Haimen, China). U0126, Tyrphostin AG1478, PP2, AG1024 and wortmannin were from Calbiochem (La Jolla, CA). Anti-HCA_1_ antibody was from Santa Cruz Biotechnology, Inc. (Santa Cruz, CA). Anti-phospho-ERK1/2, anti-ERK1/2 and anti-phospho-IGF-1R antibodies were from Cell Signaling Technology (Danvers, MA).

### Cell Culture and Transfection

CHO-K1 (ATCC# CRL-9618) cells were grown as monolayers in 50∶50 Dulbecco’s modified Eagle’s medium (DMEM): Ham’s F-12 medium containing 10% (v/v) fetal bovine serum (FBS) and glutamine (2 mM).Clonal CHO-K1 lines transfected with GPR81 or empty vector were grown in the above media, but with the addition of G418 (400 mg/L). L6 skeletal muscle cells (ATCC#CRL-1458) and HEK293 cells (ATCC# CRL-1573) were grown in DMEM supplemented with 10% (v/v) fetal bovine serum and glutamine (2 mM). Plasmid constructs were transfected or co-transfected into CHO-K1 and HEK293 cells using Lipofectamine 2000 according to the manufacturer’s instructions. All cells were incubated at 37°C in a humidified atmosphere with 5% CO2/95% air.

### Molecular Cloning and Plasmid Construction

HCA_1_ was cloned by PCR using human genomic DNA as a template. All constructs were sequenced to verify the correct sequences and orientations.

### cAMP Accumulation

After seeding in a 96-well plate overnight, stable CHO-HCA_1_ cells transfected with pCRE-Luc were grown to 90–95% confluence, stimulated with 10 μM forskolin alone or with 10 μM forskolin and different concentrations of L-lactate or 3,5-DHBA in serum-free DMEM/F12 and incubated for 4 h at 37°C. Luciferase activity was detected using a firefly luciferase kit (Promega, Madison, WI, USA). When required, cells were treated overnight with or without PTX (100 ng/mL) in serum-free DMEM/F12 before the experiment.

### Synthesis of Small Interfering RNAs and siRNA Transfection

Arrestin2 and 3 siRNAs were purchased as a SMARTpool from Dharmacon RNA Technologies (Lafayette, CO). The nonspecific control siRNA (5′-AAA CUC UAU CUG CAC GCU GAC-3′) was used as the control for all siRNA experiments. For L6 cells transfection, we followed the double hit siRNA procedure as described previously with slight modifications [12]. In brief, we seeded L6 cells at a density of 200,000 cells/6-cm dish, and after 12–16 hrs, the first siRNA transfection was performed using Lipofectamine 2000 (Invitrogen) and Opti-MEM (Invitrogen). 6–8 hrs after the first siRNA transfection, cells were split into new 6-cm dishes. Then, on Day 2, a second siRNA transfection was performed. 24 hrs after the second transfection, the cells were split for the indicated assay the following day.

### Western Blot Analysis

Cells were plated on six-well plates, grown to 80% confluence, rinsed with serum-free DMEM or DMEM/F12 (v/v) and incubated overnight in serum-free medium. For PTX treatment, the cells were pretreated with 100 ng/mL PTX overnight prior to the MAPK assay. Cells were preincubated with various inhibitors for indicated time before activation with the indicated ligands. Ligand incubation was ended by washing the cells with 2 ml of ice-cold PBS followed by the addition of RIPA lysis buffer at 4°C on a rocker for 30 min. The lysates were centrifuged at 4°C at 12,000 rpm for 15 min. The supernatants underwent electrophoresis on a 10% SDS polyacrylamide gel, which was transferred to a PVDF membrane and immunoblotted using monoclonal anti-phospho-ERK1/2 (Thr202/Tyr204) (1∶1000) or anti-phospho-IGF-1Rβ antibody (1∶500). Blots were probed with horseradish peroxidase-labeled secondary antibodies, and chemiluminescence was detected using HRP-substrate (Cell Signaling). The blots were stripped and reprobed using an anti-total ERK1/2 (1∶2000) or anti-α-tubulin monoclonal antibody as a control for protein loading. The levels of ERK 1/2 phosphorylation was normalized to total ERK1/2, and all the immunoblots were visualized and quantified by Bio-Rad Quantity One Imaging system (Bio-Rad Laboratories).

### Measurement of Receptor Internalization by Confocal Imaging

HEK-293 cells stably expressing HCA_1_-EGFP were transiently transfected with specific arrestin siRNA or a nonspecific control siRNA. After transfection (72 hrs), cells were stimulated with 20 mM lactate for 60 min. After removal of the agonist, the cells were fixed with 3% paraformaldehyde for 15 min. Confocal images were taken on a Zeiss LSM 710 microscope with an attached Axiovert 200 microscope and LSM5 computer system. Excitation was performed at 488 nm, and fluorescence detection was performed using a 525±25 nm bandpass filter. Images were collected using QED camera software and processed with Adobe Photoshop.

### Data Analysis

All results are expressed as mean ± SEM from n assays. Data was analysed using non-linear curve fitting (GraphPad PRISM version 5.0) to obtain pEC50 values. Statistical significance was determined using Student’s *t*-test. Probability values less than or equal to 0.05 were considered significant.

## Results

### Functional Expression of HCA_1_ in CHO-K1 Cells

To investigate the HCA_1_-mediated activation of extracellular signal-regulated kinases 1 and 2 (ERK1/2), we cloned human HCA_1_ and created CHO-K1 cell lines that stably expressed human HCA_1_. We first examined the functional signaling of HCA_1_ by assaying cAMP accumulation. As shown in Figs. 1a and 1b, treatment with L-lactate and 3,5-DHBA induced a ligand concentration-dependent inhibition of forskolin-stimulated cAMP increase with EC50 values of 3.58 mM and 175 μM, respectively, whereas almost no agonist-induced inhibition of the forskolin-stimulated cAMP was observed in response to L-lactate and 3,5-DHBA in parental CHO-K1 cells expressing empty vector (data not shown). The agonist-induced inhibition of the forskolin-stimulated cAMP increase could be completely blocked by pretreating with 100 ng/mL of pertussis toxin (PTX) for 16 hrs (Figs. 1a and 1b). These results suggested that HCA_1_ in stably transfected CHO-K1 cells was functional, and L-lactate and 3,5-DHBA were specific ligands for HCA_1_.

**Figure 1:** Expression and functional characterization of HCA_1_ in CHO-K1 cells. CHO-K1 cells stably expressing HCA_1_ were transfected with pCRE-Luc, cells were then stimulated with 10 μM forskolin alone or with 10 μM forskolin and different concentrations of L-lactate or 3,5-DHBA in serum-free DMEM/F12 and incubated for 4 hrs at 37°C. Luciferase activity was detected using a firefly luciferase kit (Promega, Madison, WI, USA). When required, cells were treated overnight with or without PTX (100 ng/mL) in serum-free DMEM/F12 before the experiment. All data shown are representative of at least three independent experiments. Error bars, S.E. for three replicates.

### HCA_1_ Receptors Activate ERK1/2 Signaling via MEK1/2 Following Exposure to L-lactate and 3,5-DHBA

In CHO-HCA_1_ cells, stimulation with different concentrations of agonists –L-lactate and 3,5-DHBA–evoked ERK1/2 phosphorylation in a dose-dependent manner with EC50 values of 4.05 mM, and 164 μM, respectively (Figs. 2a, 2b and 2c), whereas almost no ERK1/2 activation was observed in response to L-lactate and 3,5-DHBA in parental CHO-K1 cells expressing empty vector (Fig. 2a), which was consistent with the observation of intracellular cAMP accumulation, suggesting a specific activation of ERK1/2 via HCA_1_ by L-lactate and 3,5-DHBA. In addition, to better characterize the HCA_1_-mediated ERK1/2 signaling pathway, we also used the L6 cell line, a rat skeletal muscle cell line maybe endogenous expression of functional HCA_1_ receptors [1]. To determine whether L6 cells express endogenous HCA_1_ receptor, we used specific siRNA to knock down HCA_1_ in L6 cells. As shown in Fig. S1a, using HCA_1_ specific siRNA resulted in a significant decrease of HCA_1_ mRNA level, whereas the mRNA levels of GAPDH, did not significantly change. Moreover, the depletion of HCA_1_ resulted in a significant decrease of 3,5-DHBA-mediated ERK1/2 activation (Fig. S1b). These results demonstrated L6 cells express functional HCA_1_ receptor. So we chose L6 cells for further investigation on HCA_1_-mediated ERK1/2 activation. L6 cells were cultured in serum-free DMEM medium for 24 hrs followed by stimulation with various concentrations of 3,5-DHBA in fresh serum-free DMEM for 5 min, and the concentration-dependent activation of ERK1/2 signaling was detected with an EC50 of 4.3 mM (Fig. 2d). The HCA_1_-initiated activation of ERK1/2 was time-dependent with a maximal activation at 5 min and with a subsequent reduction to baseline by 30 min in CHO-HCA_1_ cells (Fig. 2e). A similar result was observed during 3,5-DHBA-mediated ERK1/2 activation in L6 cells (Fig. 2f).

**Figure 2:** HCA_1_ activates ERK1/2 signaling via MEK1/2 by L-Lactate and 3,5-DHBA.CHO-K1 cells expressing HCA_1_ receptor, or control parental cells harboring neither receptor, were cultured in serum-free DMEM/F-12 medium for 24 hrs. The next day, cells were then stimulated with various concentrations of L-Lactate (a and b) or 3,5-DHBA (a and c) for 5 min. (d), Serum-starved L6 cells were then stimulated with various concentrations of 3,5-DHBA for 5 min. (e), Serum-starved CHO-HCA_1_ cells were then stimulated with 10 mM L-Lactate or 300 μM 3,5-DHBA for indicated time periods. (f), Serum-starved L6 cells were then stimulated with 3 mM 3,5-DHBA for indicated time periods. Serum-starved CHO-HCA_1_ cells (g) or L6 cells (h) were pretreated with or without MEK inhibitor U0126 (1 μM) for 1 h, then stimulated with 10 mM L-Lactate or 300 μM 3,5-DHBA for CHO-HCA_1_ cells and 3 mM 3,5-DHBA for L6 cells for 5 min. The data shown are representative of at least three independent experiments. Error bars, S.E. for three replicates. Data were analyzed by using the Student’s t test (***p<0.001). IB, immunoblot; P-ERK, phospho-ERK; NS, no stimulation.

To investigate whether HCA_1_-induced ERK1/2 phosphorylation is mediated by MEK1/2 activation, the inhibitor U0126, a highly selective inhibitor of both MEK1 and MEK2, was used for the analysis of its effect on the activation of ERK1/2. As shown in Fig. 2 g, ERK1/2 activation stimulated by L-lactate and 3,5-DHBA were significantly inhibited by preincubation of CHO-HCA_1_ cells with U0126. A similar result was observed for 3,5-DHBA-mediated ERK1/2 activation in L6 cells (Fig. 2 h), which indicated that upstream MEK1/2 activation was required for HCA_1_-induced ERK1/2 phosphorylation.

### HCA_1_ Initiates ERK1/2 Activation Via the PTX-sensitive G_i_ Protein-dependent Pathway

To assess the role of the G_i_ protein in the regulation of HCA_1_-mediated activation of ERK1/2, CHO-HCA_1_ and L6 cells were cultured in the presence or absence of 100 ng/mL PTX in serum-free DMEM/F-12 or DMEM, respectively, for 24 hrs, followed by stimulation with the indicated ligand. As illustrated in Figs. 3a and 3b, the pretreatment of cells with PTX resulted in a significant inhibition of ERK1/2 phosphorylation compared to the agonist alone in both cell lines. Taken together, these data demonstrated that HCA_1_-mediated ERK1/2 pathway via a PTX-sensitive G_i_ protein-dependent mechanism.

**Figure 3:** Pertussis toxin inhibits phosphorylation of ERK1/2 induced by HCA_1_. CHO-HCA_1_ cells (a) or L6 cells (b) were cultured in serum-free DMEM/F12 or DMEM medium with or without 100 ng/ml PTX for 24 hrs, cells were then stimulated with 10 mM L-Lactate or 300 μM 3,5-DHBA for CHO-HCA_1_ for 5 min and 3 mM 3,5-DHBA for L6 cells for indicated time periods. The data shown are representative of at least three independent experiments. Error bars, S.E. for three replicates. Data were analyzed by using the Student’s t test (***p<0.001). IB, immunoblot; P-ERK, phospho-ERK; NS, no stimulation.

### Involvement of Ca^2+^ and PKC in HCA_1_-mediated ERK1/2 Activation

The pertussis toxin-sensitive G_α_ subunit can directly activate PKC, resulting in ERK1/2 phosphorylation in CHO and COS cells [13]. And our previous studies have demonstrated that PKC played an important role in HCA_2_ and HCA_3_-induced ERK1/2 activation [12], [14]. Therefore, two inhibitors of PKC were used to determine whether PKC was involved in the pathway leading to HCA_1_-mediated ERK1/2 phosphorylation. The CHO-HCA_1_ cells were pretreated with 1 μM of GF109203X (GFX) or 10 μM of Go6983 for 1 h, followed by the agonists L-lactate and 3,5-DHBA in a time course. As shown in Figs. 4a and 4b, both treatment with GF109203X and Go6983 resulted in dramatic decreases (>60%) in ERK1/2 activation. A similar result was observed during 3,5-DHBA-mediated ERK1/2 activation in L6 cells (Fig. 4c). Collectively, these data demonstrated that PKC played a determinant role in HCA_1_-mediated ERK1/2 activation.

**Figure 4:** Effects of PKC, PLC, PLD and calcium on HCA_1_-stimulated phosphorylation of ERK1/2. Serum-starved CHO-HCA_1_ cells (a and b) or L6 cells (c) were pretreated with DMSO or 10 μM Go6983 or 1 μM GF109203X (GFX) for 1 h, and then stimulated with 10 mM L-Lactate (a) or 300 μM 3,5-DHBA (b) for CHO-HCA_1_ or 3 mM 3,5-DHBA for L6 cells (c) for the indicated time periods. Serum-starved CHO-HCA_1_ cells (d and e) or L6 cells (f) were pretreated with DMSO or 20 μM U73122 or 1 μM FIPI for 1 h, and then stimulated with 10 mM L-Lactate (d) or 300 μM 3,5-DHBA (e) for CHO-HCA_1_ cells for indicated time periods, and 3 mM 3,5-DHBA for L6 cells (f) for 5 min. Serum-starved CHO-HCA_1_ cells (g) or L6 cells (h) were cultured in serum-free DMEM/F12 or DMEM media with or without EGTA (5 mM) or BAPTA-AM (50 μM) for 1 h, cells were then stimulated with 10 mM L-Lactate or 300 μM 3,5-DHBA (g) for CHO-HCA_1_ and 3 mM 3,5-DHBA for L6 cells (h) for 5 min. The data shown are representative of at least three independent experiments. Error bars, S.E. for three replicates. Data were analyzed by using the Student’s *t* test (***p<0.001). IB, immunoblot; P-ERK, phospho-ERK.

We also evaluated the effect of PLC and PLD, the upstream signaling molecules of PKC, in the HCA_1_-mediated ERK1/2 signaling pathway. The results showed that PLC inhibitor U73122 (10 μM) and PLD inhibitor FIPI (1 μM) could not block the activation of ERK1/2 induced by HCA_1_ in both CHO-HCA_1_ and L6 cells (Figs. 4d, 4e and 4f). Intriguingly, activated HCA_1_ receptors signal to ERK1/2 via PKC-dependent but PLC- and PLD-independent pathways, leading us to believe that calcium might play an important role in this process. Previous studies have shown that L-lactate causes a rapid increase of intracellular Ca^2+^ in CHO-K1 cells expressing HCA_1_ receptors [15]. Accordingly, we investigated whether or not intracellular and extracellular Ca^2+^ was involved in HCA_1_-stimulated ERK1/2 phosphorylation. Pretreatment with the extracellular Ca^2+^ chelator EGTA (5 mM) significantly inhibited ERK1/2 phosphorylation in both CHO-HCA_1_ and L6 cells (Figs. 4 g and 4 h). However, the intracellular Ca^2+^ chelator BAPTA-AM (50 μM) did not impair ERK1/2 activation by HCA_1_ receptors in both CHO-HCA_1_ and L6 cells. Taken together, the results of the present study indicated that stimulation of HCA_1_ receptors by agonists lead to ERK1/2 activation via PLC and PLD-independent and extracellular Ca^2+^ and PKC -dependent pathway.

### Involvement of PI3K and Src in HCA_1_- mediated ERK1/2 Activation

Activation of several GPCR has been shown to increase the activity of Src-family tyrosine kinases and Src has been demonstrated to be a critical regulator of GPCR activity, modulating receptor internalization, desensitization and coupling to ERK1/2 and RTK [16]. Previous studies have reported that PI3K and Src are involved in ERK1/2 activation in response to G_i_-coupled receptors [17], [18]. Our previous work also demonstrated that PI3K and Src played an important role in both HCA_2_ and HCA_3_ mediated ERK1/2 phosphorylation [12], [14]. Using CHO-HCA_1_ cells treated with the PI3K inhibitor wortmannin and the Src inhibitor PP2, we found that both wortmannin and PP2 abolished HCA_1_-stimulated ERK1/2 phosphorylation (Figs. 5a and 5b), suggesting that both PI3K and Src kinases played important roles in HCA_1_-mediated ERK1/2 activation in CHO-HCA_1_ cell lines.

**Figure 5:** Involvement of PI3K and Src in HCA_1_-mediated ERK1/2 Activation. Serum-starved CHO-HCA_1_ cells (a and b) or L6 cells (c) were pretreated with DMSO or 200 nM wortmannin or 10 μM PP2 for 1 h, and the cells were then stimulated with 10 mM L-Lactate (a) or 300 μM 3,5-DHBA (b) for CHO-HCA_1_ cells and 3 mM 3,5-DHBA for L6 cells (c) for indicated time periods. The data shown are representative of at least three independent experiments. Error bars, S.E. for three replicates. IB, immunoblot; P-ERK, phospho-ERK.

In L6 cells, pretreatment with the PI3K inhibitor wortmannin showed a similar result as seen in CHO-HCA_1_ cells (Fig. 5c). However, inhibition of Src by the selective Src kinase inhibitor PP2, did not attenuate HCA_1_-induced ERK1/2 activation in L6 cells (Fig. 5d). Taken together, these results indicated that PI3K plays an important role in HCA_1_-mediated ERK1/2 activation.

### G_βγ_ Plays a Central Role in HCA_1_-induced ERK1/2 Activation

G_βγ_ subunits bind to and activate PI3K, which is a known mediator of G_βγ_-stimulated ERK1/2 activation [17]. To test the involvement of G_βγ_-subunits in HCA_1_-mediated ERK1/2 activation, CHO-HCA_1_ and L6 cells were preincubated with G_βγ_ specific inhibitor M119K (20 μM) for 4 hrs [19], followed by stimulation with lactate or 3′5-DHBA for different lengths of time. As shown in Fig. 6, pretreatment with M119K resulted in dramatic decreases (>60%) in HCA_1_-induced ERK1/2 activation in both CHO-HCA_1_ and L6 cells, which suggested that the G_βγ_ subunit might play a central role in HCA_1_-induced ERK1/2 activation.

**Figure 6:** G_βγ_ plays a central role in HCA_1_-induced ERK1/2 activation. Serum-starved CHO-HCA_1_ cells (a and b) or L6 cells (c) were pretreated with DMSO or 20 μM M119K for 4 hrs, and the cells were then stimulated with 10 mM L-Lactate (a) or 300 μM 3,5-DHBA (b) for CHO-HCA_1_ cells and 3 mM 3,5-DHBA for L6 cells (c) for indicated time periods. The data shown are representative of at least three independent experiments. Error bars, S.E. for three replicates. IB, immunoblot; P-ERK, phospho-ERK.

### Effect of Growth Factor Receptor- Transactivation in HCA_1_-mediated ERK1/2 Activation

Many GPCRs can activate RTKs (receptor tyrosine kinases) in the absence of RTK ligands, a phenomenon called transactivation [20], [21]. Our previous studies have reported that both HCA_2_ and HCA_3_ mediated ERK1/2 activation is PDGFR transactivation-dependent in CHO cells and EGFR transactivation in A431 cells [12], [14]. Accordingly, we investigated whether PDGFR transactivation and EGFR transactivation played a role in agonist-stimulated ERK1/2 phosphorylation via HCA_1_. CHO-HCA_1_ and L6 cells were preincubated with the PDGF receptor-selective receptor tyrosine kinase inhibitor tyrphostin A9 (1 μM) for 1 h, followed by stimulation with 300 μM 3′5-DHBA for CHO-HCA_1_ cells and 3 mM 3′5-DHBA for L6 cells for different lengths of time. As shown in Figs. 7a and 7b, in CHO-HCA_1_ cells, there was only a moderate inhibition (about 25%) of HCA_1_-mediated ERK1/2 activation. In contrast, in L6 cells, there was no inhibition of ERK1/2 phosphorylation compared with cells treated with agonist alone. Lactate stimulation also exhibited a similar result in the CHO-HCA_1_ cells (Fig. 7a). As the inhibition of HCA_1_-mediated ERK1/2 activation by tyrphostin A9 was relatively small and most of the tyrphostin tyrosine kinase inhibitors were not really specific, the reduction of HCA_1_-mediated ERK1/2 phosphorylation by tyrphostin A9 was likely to be unspecific effects.

**Figure 7:** HCA_1_-induced ERK1/2 activation is dependent on insulin like growth factor-I receptor transactivation. a, Serum-starved CHO-HCA_1_ cells were pretreated with DMSO or tyrphostin A9 (1 μM) for 1 h, and then stimulated with 10 mM L-Lactate or 300 μM 3,5-DHBA for 5 min. b, Serum-starved L6 cells were pretreated with DMSO or tyrphostin A9 (1 μM) or AG1478 (1 μM) for 1 h, and then stimulated with 3 mM 3,5-DHBA for for indicated time periods. Serum-starved CHO-HCA_1_ cells (c and d) or L6 cells (e) were pretreated with DMSO or 10 μM AG1024 for 2 hrs, and the cells were then stimulated with 10 mM L-Lactate (c) or 300 μM 3,5-DHBA (d) for CHO-HCA_1_ cells and 3 mM 3,5-DHBA for L6 cells (e) for indicated time periods. f, Serum-starved L6 cells were pretreated with DMSO or PP2(10 μM) or Go6983(10 μM) or wortmannin (200 nM) for 1 h, or pretreated with M119K (20 μM) or both M119K (20 μM) and wortmannin (200 nM) for 4 hrs, and the cells were then stimulated with 5 mM 3,5-DHBA for 5 min. The data shown are representative of at least three independent experiments. Error bars, S.E. for three replicates. Data were analyzed by using the Student’s t test (*p<0.05, **p<0.01, ***p<0.001). IB, immunoblot; P-ERK, phospho-ERK.

To assess the role of EGFR transactivation in HCA_1_-induced ERK1/2 activation in cells that endogenously express HCA_1_, L6 cells were utilized for further investigation. Serum-starved L6 cells were treated with AG1478 (100 nM), an EGFR specific tyrosine kinase inhibitor, for 1 h before exposing them to 3 mM 3,5-DHBA. As shown in Fig. 7b, AG1478 pretreatment have no inhibition of ERK1/2 phosphorylation compared with cells treated with agonist alone.

Previous studies have demonstrated that Src can regulate IGF-I receptor [22], and Src kinase can substitute for the receptor kinase in phosphorylating and activating IGF-I receptor [23]. Next, we investigate whether IGF-1R transactivation was involved in HCA_1_-mediated ERK1/2 activation. CHO-HCA_1_ and L6 cells were preincubated with a selective insulin like growth factor-I (IGF-I) receptor tyrosine kinase inhibitor tyrphostin AG 1024 (10 μM) for 2 hrs, followed by stimulation with 300 μM 3′5-DHBA for CHO-HCA_1_ cells and 3 mM 3′5-DHBA for L6 for different lengths of time. As shown in Figs. 7d and 7e, in both AG1024 pretreated CHO-HCA_1_ and L6 cells, ERK1/2 phosphorylation was decreased over 50% compared with cells treated with agonist alone. Lactate stimulation also exhibited similar results in CHO-HCA_1_ cells (Fig. 7c), showing that IGF-1R transactivation is involved in HCA_1_-induced ERK1/2 activation in both CHO-HCA_1_ and L6 cells.

To further determine whether HCA_1_ can activate IGF-1R, L6 cells were treated with 3,5-DHBA for 5 min, as shown in Fig7f, 3,5-DHBA treatment induced about two fold IGF-1R phosphorylation. Pretreatment with PP2 inhibitor resulted in moderate decreases (about 15%) in HCA_1_-induced IGF-1R activation. However, M119K or wortmannin pretreatment resulted in more notable decreases (40 and 55% respectively) in HCA_1_-mediated IGF-1R phosphorylation, simultaneous inhibition of G_βγ_ and PI3K resulted in a nearly complete inhibition of IGF-1R phosphorylation (fig. 7f), suggesting the involvement of G_βγ_ and PI3K in HCA_1_-mediated IGF-1R phosphorylation.

### Arrestin3 is Involved in HCA_1_ Internalization, but Arrestins are not Involved in HCA_1_-mediated ERK1/2 Activation

To evaluate the role of arrestins in the regulation of HCA_1_ internalization and ERK1/2 activation, we used specific siRNAs to reduce the expression of arrestin2 and arrestin3 in HEK-293 cells stably expressing HCA_1_ receptors. The endogenous expression of arrestins was effectively and specifically knocked-down by specific siRNA treatment but was unaffected in cells treated with non-specific or control siRNAs (Fig. 8a). Silencing arrestin3 effectively inhibited HCA_1_ internalization, whereas knock-down of arrestin2 had no effect on the internalization of HCA_1_ receptors (Fig. 8b). We further investigated the effect of knock-down of arrestins on ERK1/2 activation, and no difference was observed between control and knock-down cells (Fig. 8c). Taken together, arrestin3 might be involved in HCA_1_ receptor internalization, but both arrestins were not required for HCA_1_-mediated ERK1/2 activation.

**Figure 8:** There is no involvement of arrestins in HCA_1_-mediated ERK1/2 activation. a, HEK-293 cells stably expressing HCA_1_ were transfected with specific arrestin siRNA or a nonspecific control siRNA, 72 hrs after transfection, cells were harvested, and equal amounts of total cellular lysate were separated by 10% SDS-PAGE, transferred to a PVDF membrane, and incubated with anti-arrestin2/3 antibody. b, HEK-293 cells stably expressing HCA_1_-EGFP were transfected with specific arrestin siRNA or a non-specific control siRNA,72 hrs after transfection, cells were stimulated with 20 mM lactate for 60 min and examined with confocal microscopy as described under ‘Experimental Procedures.’ c, 72 hrs after transfection with specific arrestin siRNA or non-specific control siRNA, cells were stimulated with 20 mM lactate for the indicated time periods and immunoblotted using monoclonal anti-phospho-MAPK E10 (Thr202/Tyr204), and then the blots were stripped and reprobed for total ERK1/2 to control for loading. The data and pictures shown are representative of at least three independent experiments. Error bars, S.E. for three replicates. Data were analysed by Student’s *t* test (***P<0.001).

## Discussion

Lactate is an important metabolic intermediate released by skeletal muscle and other organs including the adipose tissue, which converts glucose into lactate under the influence of insulin [5]. Two recent studies showed that lactate was the endogenous ligand of hydroxy-carboxylic acids (HCAs) receptor 1 [1], [15]. And lactate was a specific agonist of HCA_1_ as it did not activate the closely related receptors HCA_2_ and HCA_3_. Activation of HCA_1_ in adipocytes by lactate results in the inhibition of lipolysis at physiologically relevant lactate concentrations (1 to 20 mM) [1], suggesting that HCA_1_ could be a new target for dyslipidemia treatment without the unwanted side effect of cutaneuous flushing. As a metabolite of glucose, lactate concentrations rise in vivo following a glucose load [1], and thus HCA_1_ may also serve a regulatory role for glucose metabolism. It has been suggested that lactate plays a role in insulin signaling, particularly in insulin mediated anti-lipolytic effects [5]. It has also been suggested that HCA_1_ may play a role in muscle glucose and fatty acid metabolism [6]. However, the underlying molecular mechanisms for HCA_1_ signaling remain largely unknown. In the current study, we focused on a detailed characterization of HCA_1_-mediated MAPK signalling pathways.

In the present study, the CHO-K1 cell line was selected as a cellular model system for characterizing HCA_1_ receptor signaling pathways as it was a commonly used cell line for investigating GPCR coupling to various signaling pathways. For better delineation of HCA_1_-mediated phosphorylation of ERK1/2, we also used L6 cell line, a rat skeletal muscle cell line, which endogenously expressed rat HCA_1_ receptors, in our current study. The HCA_1_ receptor was a G_i_ protein-coupled receptor, upon stimulation by agonists, HCA_1_ receptors triggered an inhibitory effect on adenylate cyclase that led to a decrease of intracellular cAMP levels in a PTX-sensitive manner (Figs. 1a and 1b). Additionally, both CHO-K1 stably expressing HCA_1_ and L6 cell lines showed a time-dependent activation of ERK1/2 in response to L-lactate or 3′5-DHBA, peaking at approximately 5 min and returning to basal levels at 30 min, however, the activation of ERK1/2 was significantly attenuated in the presence of PTX (Figs. 3a and 3b). These results indicated that the essential involvement of a heterotrimeric G_i_ protein in ERK1/2 phosphorylation at an early stage was common to both CHO and L6 cells.

Previous studies have shown that L-lactate causes a rapid increase of intracellular Ca^2+^ in CHO-K1 cells expressing HCA_1_ receptors [16]. We next evaluated the role of PKC in the regulation of HCA_1_-induced ERK1/2 phosphorylation using specific inhibitors. Our present data demonstrated that the HCA_1_-induced ERK1/2 activation was blocked by Go6983 and GF109203x, PKC inhibitors, suggesting that the PKC pathway participates in ERK1/2 activation (Figs. 4a, 4b and 4c). The involvement of PLC and PLD as a contributor to HCA_1_-mediated ERK1/2 activation was assessed by incubating cells with a PLC inhibitor, U73122 or a PLD inhibitor FIPI. Our results shown that both U73122 and FIPI exhibited no significant inhibition of ERK1/2 phosphorylation by activated HCA_1_ (Figs. 4d, 4e and 4f). Furthermore, we found that HCA_1_-induced ERK1/2 activation was abolished by the depletion of extracellular Ca^2+^ by the chelator EGTA but not by BAPTA-AM, an intracellular Ca^2+^ chelator in both CHO-HCA_1_ and L6 cells, suggesting that Ca^2+^ channel may play an important part in HCA_1_-mediated ERK1/2 activation (Figs. 4 g and 4 h). Taken together, these data suggested the involvement of extracellular Ca^2+^ and PKC in HCA_1_-mediated ERK1/2 activation.

Moreover, phosphatidylinositol-3′ kinases (PI3K) and Src family non-receptor tyrosine kinases have each been proposed as early intermediates in the pathway to induce EGF receptor transactivation [24], [25]. In the present study, we observed that PI3K involved in IGF-1R transactivated phosphorylation of ERK1/2, whereas the Src kinase was not required for HCA_1_-induced IGF-1R transactivation in L6 cells.

There is a growing body of evidence to suggest that the transactivation of growth factor receptors is another mechanism by which GPCRs mediate ERK1/2 phosphorylation [20]. Our previous study demonstrated that, in CHO-K1 cells, both HCA_2_ and HCA_3_-mediated ERK1/2 activation was potently inhibited by the PDGF receptor-selective inhibitor tyrphostin A9, and in A431 cells, the EGF receptor-selective inhibitor AG1478 was found to significantly impair ERK1/2 activation. Our present research showed that PDGFR and EGFR were well possible playing no role in HCA_1_-induced ERK1/2 phosphorylation in CHO-K1 and L6 cells. In contrast, HCA_1_-mediated ERK1/2 phosphorylation was found to be significantly impaired by AG1024, an insulin-like growth factor-1 receptor specific tyrosine kinase, in both two cell lines. These results suggested that a transactivation of insulin-like growth factor-1 receptor participateed in HCA_1_-mediated ERK1/2 phosphorylation. Previous study also have shown that the insulin-like growth factor-1 receptor can be transactivated in response to GPCR ligands such as thrombin [26] and angiotensin II [27].

In addition, we observed that pretreated the cells with M119K, an inhibitor of G_βγ_ subunit-dependent signaling [19], effectively attenuated the IGF-1R receptor phosphorylation and ERK1/2 activation triggered by HCA_1_(Figs. 6a, 6b and 6c). Simultaneous inhibition of G_βγ_ and PI3K resulted in a nearly complete inhibition of IGF-1R phosphorylation. These results indicated that G_βγ_ subunit might act as an early signal mediating HCA_1_-induced IGF-1R receptor transactivation. The major effects of G_i_ activation on ERK1/2 cascade appear to be mediated via its G_βγ_ subunits [28], [29]. Previous studies have shown that G_i_-type GPCRs stimulate Ca^2+^ mobilization through the binding of G_βγ_ subunits to PLC [30], [31]. It has also been reported that the best understood mechanism whereby the G_βγ_ subunits stimulate ERK1/2 is through the ‘transactivation’ of classical receptor tyrosine kinases, e.g., the EGF and platelet-derived growth factor (PDGF) receptors [21]. Thus, we postulated that upon stimulation of HCA_1_ by agonists, activated G_i_ protein impaired cAMP production and released G_βγ_ subunits, the free G_βγ_ subunits caused IGF-1R transactivation.

Arrestins are traditionally recognized as playing a well-established role in the termination of receptor-G-protein coupling and the initiation of clathrin-dependent internalization [32]. However, there is a growing body of evidence indicates that arrestins function as signal transducers for many GPCRs to mediate ERK1/2 activation [33]. Arrestins are required for later phase activation of the ERK1/2 pathway mediated by angiotensin II type 1A (AT1A) [34], β2-adrenergic [35], vasopressin 2 [36], and parathyroid hormone (PTH) [37] receptors, whereas, in the dopamine D2 and D3 receptor [38] and the formyl peptide receptor (FPR) [39], arrestins have been found to play no role or only a minor role in the activation of the ERK1/2 pathway. Our results using siRNA showed that arrestin3 was required for agonist-mediated HCA_1_ internalization, whereas knockdown of arrestin2 or arrestin3 using siRNA had no effect on ERK1/2 activation. These results were in good agreement with our previous observation for the HCA_2_-mediated activation of the ERK1/2 pathway [40].

In conclusion, we have characterized the molecular mechanisms of HCA_1_-mediated activation of the ERK1/2 pathway and demonstrated that the G_βγ_ subunit dissociated from the activated G_i_ protein played a central role in the regulation of HCA_1_-activated ERK1/2 phosphorylation via PKC pathway activation and IGF-1R transactivation. Furthermore, we found arrestin-2 and arrestin-3 had no effect on HCA_1_-mediated ERK1/2 activation by using arrestin-2/3 specific siRNA, whereas HCA_1_ internalization was arrestin3-dependent. However, additional investigations will be necessary to further clarify the role of the ERK1/2 pathway in HCA_1_-mediated insulin-dependent inhibition of lipolysis.

## Supporting Information

Figure S1 a, L6 cells were transfected with specific HCA1 siRNA or a nonspecific control siRNA (The HCA1 siRNA sequence was 5′- ACCUGGAAGUCGAGCACUA -3′, whereas 5′-AAACUCUAUCUGCACGCUGAC-3′ was used for nonspecific control). A total of 96 hrs after transfection, cells were harvested, mRNA levels of GAPDH and HCA1 were measured by quantitative real-time–PCR. b, A total of 96 hrs after transfection with specific HCA1 siRNA or nonspecific control siRNA, L6 cells were stimulated with DMSO or 3 mM 3,5-DHBA for 5 min and immunoblotted using monoclonal anti- phospho-MAPK E10 (Thr202/Tyr204), and then the blots were stripped and reprobed for total ERK to control for loading. The data shown are representative of at least three independent experiments. Error bars, S.E. for three replicates. Data were analyzed by using the Student’s t test (***p<0.001). IB, immunoblot; P-ERK, phospho-ERK.
(TIF)

## References

[1] LiuC, WuJ, ZhuJ, KueiC, YuJ, et al (2009) Lactate inhibits lipolysis in fat cells through activation of an orphan G-protein-coupled receptor, GPR81. J Biol Chem 284: 2811–2822.1904706010.1074/jbc.M806409200

[2] TaggartAK, KeroJ, GanX, CaiTQ, ChengK, et al (2005) (D)-beta-Hydroxybutyrate inhibits adipocyte lipolysis via the nicotinic acid receptor PUMA-G. J Biol Chem 280: 26649–26652.1592999110.1074/jbc.C500213200

[3] AhmedK, TunaruS, LanghansCD, HansonJ, MichalskiCW, et al (2009) Deorphanization of GPR109B as a receptor for the beta-oxidation intermediate 3-OH-octanoic acid and its role in the regulation of lipolysis. J Biol Chem 284: 21928–21933.1956106810.1074/jbc.M109.019455PMC2755917

[4] AhmedK, TunaruS, OffermannsS (2009) GPR109A, GPR109B and GPR81, a family of hydroxy-carboxylic acid receptors. Trends Pharmacol Sci 30: 557–562.1983746210.1016/j.tips.2009.09.001

[5] AhmedK, TunaruS, TangC, MullerM, GilleA, et al (2010) An autocrine lactate loop mediates insulin-dependent inhibition of lipolysis through GPR81. Cell Metab 11: 311–319.2037496310.1016/j.cmet.2010.02.012

[6] GeH, WeiszmannJ, ReaganJD, GupteJ, BaribaultH, et al (2008) Elucidation of signaling and functional activities of an orphan GPCR, GPR81. J Lipid Res 49: 797–803.1817460610.1194/jlr.M700513-JLR200

[7] LorenzK, SchmittJP, SchmitteckertEM, LohseMJ (2009) A new type of ERK1/2 autophosphorylation causes cardiac hypertrophy. Nat Med 15: 75–83.1906090510.1038/nm.1893

[8] SunY, ChengZ, MaL, PeiG (2002) Beta-arrestin2 is critically involved in CXCR4-mediated chemotaxis, and this is mediated by its enhancement of p38 MAPK activation. J Biol Chem 277: 49212–49219.1237018710.1074/jbc.M207294200

[9] SchwindingerWF, RobishawJD (2001) Heterotrimeric G-protein betagamma-dimers in growth and differentiation. Oncogene 20: 1653–1660.1131391310.1038/sj.onc.1204181

[10] AhnS, KimJ, HaraMR, RenXR, LefkowitzRJ (2009) {beta}-Arrestin-2 Mediates Anti-apoptotic Signaling through Regulation of BAD Phosphorylation. J Biol Chem 284: 8855–8865.1917193310.1074/jbc.M808463200PMC2659243

[11] PuJ, PengG, LiL, NaH, LiuY, et al (2011) Palmitic acid acutely stimulates glucose uptake via activation of Akt and ERK1/2 in skeletal muscle cells. J Lipid Res 52: 1319–1327.2151869610.1194/jlr.M011254PMC3122917

[12] LiG, DengX, WuC, ZhouQ, ChenL, et al (2011) Distinct kinetic and spatial patterns of protein kinase C (PKC)- and epidermal growth factor receptor (EGFR)-dependent activation of extracellular signal-regulated kinases 1 and 2 by human nicotinic acid receptor GPR109A. J Biol Chem 286: 31199–31212.2176809310.1074/jbc.M111.241372PMC3173092

[13] van BiesenT, HawesBE, RaymondJR, LuttrellLM, KochWJ, et al (1996) G(o)-protein alpha-subunits activate mitogen-activated protein kinase via a novel protein kinase C-dependent mechanism. J Biol Chem 271: 1266–1269.857610910.1074/jbc.271.3.1266

[14] Zhou Q, Li G, Deng X, H X, Chen L, et al.. (2012) Activated Human Hydroxy-Carboxylic Acid Receptor-3 Signals to MAP Kinase Cascades via the PLC-Dependent PKC and MMP-Mediated EGFR Pathways. Br J Pharmacol.10.1111/j.1476-5381.2012.01875.xPMC340280222289163

[15] CaiTQ, RenN, JinL, ChengK, KashS, et al (2008) Role of GPR81 in lactate-mediated reduction of adipose lipolysis. Biochem Biophys Res Commun 377: 987–991.1895205810.1016/j.bbrc.2008.10.088

[16] LuttrellDK, LuttrellLM (2004) Not so strange bedfellows: G-protein-coupled receptors and Src family kinases. Oncogene 23: 7969–7978.1548991410.1038/sj.onc.1208162

[17] Lopez-IlasacaM, CrespoP, PelliciPG, GutkindJS, WetzkerR (1997) Linkage of G protein-coupled receptors to the MAPK signaling pathway through PI 3-kinase gamma. Science 275: 394–397.899403810.1126/science.275.5298.394

[18] KranenburgO, VerlaanI, HordijkPL, MoolenaarWH (1997) Gi-mediated activation of the Ras/MAP kinase pathway involves a 100 kDa tyrosine-phosphorylated Grb2 SH3 binding protein, but not Src nor Shc. EMBO J 16: 3097–3105.921462710.1093/emboj/16.11.3097PMC1169928

[19] KiruiJK, XieY, WolffDW, JiangH, AbelPW, et al (2010) Gbetagamma signaling promotes breast cancer cell migration and invasion. J Pharmacol Exp Ther 333: 393–403.2011037810.1124/jpet.109.164814PMC2872950

[20] PierceKL, LuttrellLM, LefkowitzRJ (2001) New mechanisms in heptahelical receptor signaling to mitogen activated protein kinase cascades. Oncogene 20: 1532–1539.1131389910.1038/sj.onc.1204184

[21] GschwindA, ZwickE, PrenzelN, LesererM, UllrichA (2001) Cell communication networks: epidermal growth factor receptor transactivation as the paradigm for interreceptor signal transmission. Oncogene 20: 1594–1600.1131390610.1038/sj.onc.1204192

[22] BromannPA, KorkayaH, CourtneidgeSA (2004) The interplay between Src family kinases and receptor tyrosine kinases. Oncogene 23: 7957–7968.1548991310.1038/sj.onc.1208079

[23] PetersonJE, KulikG, JelinekT, ReuterCW, ShannonJA, et al (1996) Src phosphorylates the insulin-like growth factor type I receptor on the autophosphorylation sites. Requirement for transformation by src. J Biol Chem 271: 31562–31571.894017310.1074/jbc.271.49.31562

[24] LinAL, ZhuB, ZhangW, DangH, ZhangBX, et al (2008) Distinct pathways of ERK activation by the muscarinic agonists pilocarpine and carbachol in a human salivary cell line. Am J Physiol Cell Physiol 294: C1454–1464.1838529010.1152/ajpcell.00151.2007

[25] Lopez-IlasacaM, GutkindJS, WetzkerR (1998) Phosphoinositide 3-kinase gamma is a mediator of Gbetagamma-dependent Jun kinase activation. J Biol Chem 273: 2505–2508.944655010.1074/jbc.273.5.2505

[26] DuJ, BrinkM, PengT, MottironiB, DelafontaineP (2001) Thrombin regulates insulin-like growth factor-1 receptor transcription in vascular smooth muscle: characterization of the signaling pathway. Circ Res 88: 1044–1052.1137527410.1161/hh1001.090840

[27] ZahradkaP, LitchieB, StorieB, HelwerG (2004) Transactivation of the insulin-like growth factor-I receptor by angiotensin II mediates downstream signaling from the angiotensin II type 1 receptor to phosphatidylinositol 3-kinase. Endocrinology 145: 2978–2987.1497614810.1210/en.2004-0029

[28] HawesBE, van BiesenT, KochWJ, LuttrellLM, LefkowitzRJ (1995) Distinct pathways of Gi- and Gq-mediated mitogen-activated protein kinase activation. J Biol Chem 270: 17148–17153.761551010.1074/jbc.270.29.17148

[29] CrespoP, XuN, SimondsWF, GutkindJS (1994) Ras-dependent activation of MAP kinase pathway mediated by G-protein beta gamma subunits. Nature 369: 418–420.819677010.1038/369418a0

[30] DickensonJM, HillSJ (1998) Involvement of G-protein betagamma subunits in coupling the adenosine A1 receptor to phospholipase C in transfected CHO cells. Eur J Pharmacol 355: 85–93.975494210.1016/s0014-2999(98)00468-3

[31] DornGW2nd, OswaldKJ, McCluskeyTS, KuhelDG, LiggettSB (1997) Alpha 2A-adrenergic receptor stimulated calcium release is transduced by Gi-associated G(beta gamma)-mediated activation of phospholipase C. Biochemistry. 36: 6415–6423.10.1021/bi970080s9174358

[32] LuttrellLM, LefkowitzRJ (2002) The role of beta-arrestins in the termination and transduction of G-protein-coupled receptor signals. J Cell Sci 115: 455–465.1186175310.1242/jcs.115.3.455

[33] LefkowitzRJ, ShenoySK (2005) Transduction of receptor signals by beta-arrestins. Science 308: 512–517.1584584410.1126/science.1109237

[34] AhnS, WeiH, GarrisonTR, LefkowitzRJ (2004) Reciprocal regulation of angiotensin receptor-activated extracellular signal-regulated kinases by beta-arrestins 1 and 2. J Biol Chem 279: 7807–7811.1471182410.1074/jbc.C300443200

[35] ShenoySK, DrakeMT, NelsonCD, HoutzDA, XiaoK, et al (2006) beta-arrestin-dependent, G protein-independent ERK1/2 activation by the beta2 adrenergic receptor. J Biol Chem 281: 1261–1273.1628032310.1074/jbc.M506576200

[36] RenXR, ReiterE, AhnS, KimJ, ChenW, et al (2005) Different G protein-coupled receptor kinases govern G protein and beta-arrestin-mediated signaling of V2 vasopressin receptor. Proc Natl Acad Sci U S A 102: 1448–1453.1567118010.1073/pnas.0409534102PMC547876

[37] Gesty-PalmerD, ChenM, ReiterE, AhnS, NelsonCD, et al (2006) Distinct beta-arrestin- and G protein-dependent pathways for parathyroid hormone receptor-stimulated ERK1/2 activation. J Biol Chem 281: 10856–10864.1649266710.1074/jbc.M513380200

[38] BeomS, CheongD, TorresG, CaronMG, KimKM (2004) Comparative studies of molecular mechanisms of dopamine D2 and D3 receptors for the activation of extracellular signal-regulated kinase. J Biol Chem 279: 28304–28314.1510284310.1074/jbc.M403899200

[39] GripentrogJM, MiettinenHM (2008) Formyl peptide receptor-mediated ERK1/2 activation occurs through G(i) and is not dependent on beta-arrestin1/2. Cell Signal 20: 424–431.1806074110.1016/j.cellsig.2007.11.002PMC2330276

[40] LiG, ShiY, HuangH, ZhangY, WuK, et al (2010) Internalization of the human nicotinic acid receptor GPR109A is regulated by G(i), GRK2, and arrestin3. J Biol Chem 285: 22605–22618.2046038410.1074/jbc.M109.087213PMC2903394

